# Comparative Insights into the Skin Beneficial Properties of Probiotic *Lactobacillus* Isolates of Skin Origin

**DOI:** 10.1155/2022/7728789

**Published:** 2022-05-13

**Authors:** Hye-Won Lim, Yu-Hua Huang, Gyuri Kyeong, Minsik Park, Chang-Jin Lim

**Affiliations:** ^1^R&D Center, Shebah Biotech Inc., G-Tech Village, Chuncheon 24398, Republic of Korea; ^2^Department of Molecular and Cellular Biochemistry, Kangwon National University School of Medicine, Chuncheon 24341, Republic of Korea; ^3^Department of Biochemistry, Kangwon National University, Chuncheon 24341, Republic of Korea

## Abstract

In recent times, probiotics have been emerging as one of valuable cosmetic resources. This work was undertaken to evaluate and compare the skin beneficial properties of three *Lactobacillus* strains, namely, *L. plantarum* SB202, *L. fermentum* SB101, and *L. paraplantarum* SB401, originally isolated from the healthy skins of Koreans. The *Lactobacillus* isolates were individually grown in MRS broth, and the corresponding cell-free conditioned mediums (CMs), LP202, LF101 and LPP401, were prepared for analyzing diverse cosmetic potentials at a comparative perspective. The superoxide radical and nitrite ion scavenging activities of the CMs were in the orders of LPP401 ≥ LF101 > LP202 and LPP401 > LF101≒LPP202, respectively. They attenuated the lipopolysaccharide-induced reactive oxygen species (ROS) and nitrite ion levels in RAW264.7 murine macrophages both in the order of LPP401 ≥ LF101 > LP202, implying their anti-inflammatory properties. They exhibited antityrosinase activities in the order of LPP401 > LF101 ≥ LP202 and diminished *α*-melanocyte-stimulating hormone-induced melanin levels in B16F10 melanoma cells in the order of LPP401≒LF101 > LP202, suggesting their skin whitening activities. They enhanced cornfield envelope formation in HaCaT keratinocytes in the order of LPP401 > LF101 > LP202. They inhibited the in vitro hyaluronidase and elastase activities in the orders of LPP401 > LP202 ≥ LF101 and LPP401 ≥ LP202 > LF101, respectively. Their enhancing properties on the synthesis of procollagen type I in normal human dermal fibroblasts were in the order of LF101≒LPP401 > >LP202. The CMs possess various cosmetic characteristics, such as antioxidant, skin whitening, antiaging, barrier improving, and anti-inflammatory activities. LPP401, the CM prepared from *L. paraplantarum* SB401, has been evaluated to be more desirable cosmetic resource than LP202 and LF101.

## 1. Introduction

Probiotics (or “probiotic” microorganisms), defined as live microorganisms such as bacteria and fungi which confer health benefits on the host organisms in adequate amounts, have become increasingly popular during the past few decades due to extensively broadening the related scientific information. Major action mechanisms of probiotics presently include enhancement of epithelial barrier, alteration of gastrointestinal microbiota, induction of apoptosis, increased adhesion to intestinal mucosa, competition with potential pathogens for nutrients or adhesion sites, degradation of toxins, enhancement of immune response, and production of antimicrobial substances [1, 2]. Even some nonviable probiotics and their components, or so-called paraprobiotics, have been known to possess probiotic characteristics. The most commonly known types of prebiotics, which are capable of inducing the growth and activity of probiotics, are oligosaccharides, inulin-type fructan, sugar alcohols, and complex polysaccharides such as cellulose and *β*-glucan^3^. The health benefits of synbiotics, meaning, a combination of probiotics and prebiotics, are being also under recent interest. Lactic acid bacteria (LAB), a heterogeneous group of Gram-positive bacteria which receive generally recognized as safe (GRAS) status, are the most well-known probiotics. *Lactobacillus* and *Bifidobacterium* (earlier collectively referred as to *Lactobacillus bifidus*), belonging to LAB, are the very widely used probiotic genera which were originally isolated from the human gastrointestinal tracts.

Probiotics have been shown to have varied skin beneficial properties such as mediation of skin inflammation, treatment of various skin diseases, prevention of allergic contact dermatitis, decolonization of skin pathogens, and treatment against skin pathogens [3]. They also play crucial roles in balancing the good bacteria that reside within the skin, strengthening the skin barrier, promoting better moisture adsorption, and aiding in delaying the signs of skin aging [4]. Probiotic bacteriotherapy has been suggested to have diverse potentials in preventing and treating the skin diseases including atopic dermatitis, acne and eczema, in skin hypersensitivity, wound protection and UV-induced skin damage, and as a cosmetic resource [5].

The probiotic species *L. plantarum*, *L. fermentum*, and *L. paraplantarum* have been assessed to have skin-targeting beneficial effects, when live or killed cells, cellular lysates or conditioned media (supernatants) were administered either topically or orally. *L. plantarum* possesses skin anticancer, skin antiphotoaging, skin antiaging, wound healing, immunity-promoting, and whitening properties [6–11]. *L. fermentum* exhibits antioxidant, gut barrier function improving, and skin antiphotoaging properties [12–14]. In particular, *L. fermentum* ATCC 23271 strongly displays a higher inhibitory activity against *Candida* spp. associated to vaginal candidiasis in comparison to other well-characterized *Lactobacillus* species, including *L. plantarum*, *L. acidophilus*, and *L. rhamnosus* [15]. *L. paraplantarum* was verified to possess antifungal, antioxidant, immunostimulatory, antihyperalgesic, and antiedematous properties [16–18].

In the present work, the skin beneficial properties of three *Lactobacillus* isolates, *L. plantarum* SB202, *L. fermentum* SB101, and *L. paraplantarum* SB401, indigenous to Korean skins were assessed at a comparative perspective.

## 2. Materials and Methods

### 2.1. Chemicals

Ascorbic acid (AA), arbutin (AR), bovine serum albumin (BSA), dimethyl sulfoxide (DMSO), phosphate-buffered saline (PBS), sodium nitrite, 3-(4,5-dimethylthiazol-2-yl)-2,5-diphenyltetrazolium bromide (MTT), 2′,7′-dichlorodihydrofluorescein diacetate (DCFH-DA), lipopolysaccharide (LPS), NADH, nitroblue tetrazolium, phenazine methosulfate, dithiothreitol (DTT), mushroom tyrosinase, L-3,4-dihydroxyphenylalanine (L-DOPA), Griess reagent, *α*-melanocyte stimulating hormone (*α*-MSH), bovine testes hyaluronidase, hyaluronan (HA), porcine pancreatic elastase, and *N*-succinyl-(L-Ala)_3_-*p*-nitroanilide (STANA) were from Sigma-Aldrich Chemical Co. (St Louis, MO, USA). All other chemicals used were of the relatively high grade commercially available.

### 2.2. Bacterial Cell Growth

The three *Lactobacillus* isolates of Korean skin origin, *Lactobacillus plantarum* SB202 (KCTC 14087BP, Korean Collection for Type Cultures, Korea Research Institute of Bioscience and Biotechnology, Republic of Korea), *Lactobacillus fermentum* SB101 (KCTC 14086BP, Korean Collection for Type Cultures), and *Lactobacillus paraplantarum* SB401 (KCTC 14088BP, Korean Collection for Type Cultures), were grown in de Man, Rogosa, and Sharpe (MRS) medium at 37°C.

### 2.3. Preparation of Bacterial Conditioned Mediums (CMs)

The isolated single colonies, picked from MRS agar plates, were subjected to main cultures in MRS broth at 37°C after three subcultures. After the 5-day incubation, the CMs were obtained from the bacterial cultures through centrifugation, sterilized using 0.2 *μ*m pore size membrane filters, and named LP202, LF101, and LPP401 for *L. plantarum* SB202, *L. fermentum* SB101, and *L. paraplantarum* SB401 cultures, respectively. When CMs were comparatively used, the experimental values were normalized to those obtained with the *Lactobacillus* cultures grown up to an absorbance of 8.0 at 600 nm. If necessary, MRS medium itself was used in parallel with the cell-free CMs containing the residual MRS medium ingredients after the bacterial growth plus the products or metabolites extracellularly released from the corresponding *Lactobacillus* cells during the growth.

### 2.4. Mammalian Cell Growth

Mammalian cell lines (ATCC, Manassas, VA, USA), such as RAW264.7 murine macrophages, an immortalized human keratinocyte HaCaT cell line, and a murine melanoma cell line B16F10, were grown in Dulbecco's Modified Eagle's Medium (DMEM) containing 10% heat-inactivated fetal bovine serum (FBS), 100 *μ*g/mL streptomycin, and 100 units/mL penicillin in a humidified atmosphere with 5% CO_2_ at 37°C. An additional mammalian cell line, normal human dermal fibroblast (NHDF) cells (PromoCell GmbH, Heidelberg, Germany) were cultured in Fibroblast Growth Medium-2 (Lonza Group AG, Basel, Switzerland) with 2% FBS, 0.4% insulin, 0.4% human fibroblast growth factor-basic, and 0.4% gentamicin in the same growth conditions. Prior to the treatments in typical procedures, 1 × 10^5^ cells, seeded on 24- or 6-well plates, were grown overnight and two times washed with 1 mL PBS and suspended in 1 mL FBS-free medium. The mammalian cells were then subjected to appropriate treatments.

### 2.5. Cellular Viability Assay

To measure the cytotoxicity of CMs, under experimental conditions, on the cultured mammalian cells, the cellular viabilities were determined using an MTT assay which is used to assess metabolic activity [19]. Cultured cells were treated with the CMs (10 *μ*L) for 1 h and then washed out. The medium was suctioned out, and the cells were treated with 5 *μ*g/mL MTT for 4 h. The purple formazan crystals, produced with the reduction of MTT in the mitochondria of living cells, were dissolved in DMSO. The amount of formazan was quantitated by the absorbance at 540 nm.

### 2.6. In Vitro Superoxide Radical Scavenging Activity Assay

As previously described [20], the in vitro superoxide radical scavenging activity of the CMs was determined. In brief, CM (10 *μ*L) was added to 180 *μ*L of 1 mM Tris buffer (pH 8.0) with 156 *μ*M NADH, 100 *μ*M nitroblue tetrazolium, and 20 *μ*M phenazine methosulfate. The reaction mixture was kept for 5 min at 25°C. The absorbance at 560 nm was measured at a microplate reader.

### 2.7. In Vitro Nitrite Scavenging Activity Assay

The in vitro nitrite scavenging activity of the CMs was determined as previously described [21]. Briefly, CM (10 *μ*L) was mixed with 30 *μ*L of 0.1 mM citrate buffer (pH 3.0) and 6 *μ*L of 50 *μ*g/mL sodium nitrite. The reaction mixture was kept at 37°C for 60 min and then mixed with the equal volume of Griess reagent. After 10 min incubation, the absorbance at 538 nm was measured using a microplate reader.

### 2.8. Determination of Intracellular ROS in Macrophages

A fluorescent probe DCFH-DA, which produces 2′,7′-dichlorofluorescein (DCF; *λ*_excitation_ = 485 nm, *λ*_emission_ = 530 nm) upon enzymatic reduction and subsequent oxidation by ROS, was used [22]. After the preincubation with CM (10 *μ*L) for 1 h, the cultured macrophages were treated for 24 h with 10 *μ*g/mL LPS. The cells were incubated with 5 *μ*M DCFH-DA for 30 min at 37°C and harvested. They were twice washed with 1 mL FBS-free DMEM and suspended in 1 mL FBS-free DMEM. The intracellular ROS levels were quantitated by measuring the fluorescence at a multimode microplate reader (Synergy™ Mx, BioTek Instruments, Winooki, VT, USA).

### 2.9. Determination of Nitrite in Macrophage Culture Supernatants

Accumulated nitrite ions (NO_2_^−^), an index of cell-released NO, in macrophage culture supernatants were quantitated using a spectrophotometric assay based upon Griess reaction [21], which was similar to the protocol described in “2.7. In vitro Nitrite Scavenging Activity Assay” in Materials and Methods. An equal volume of Griess reagent was reacted with culture supernatant, obtained from the macrophage cultures treated with 10 *μ*L CM, for 10 min at 25°C, and the absorbance at 538 nm was measured using a microplate reader. The calibration curve was constructed using known concentrations (0–150 *μ*M) of sodium nitrite.

### 2.10. Antityrosinase Activity Assay

As previously described [23], the L-DOPA oxidation activity of tyrosinase was determined. Each reaction mixture (200 *μ*L) contained 0.04 mM phosphate buffer (pH 6.8), 0.5 mM L-DOPA, CM (10 *μ*L), and 6 units/mL mushroom tyrosinase and was then incubated at 37°C for 10 min. The amount of dopaquinone produced was determined by the change in the absorbance at 450 nm using a plate reader.

### 2.11. Determination of Melanin Content in Melanoma Cells

As previously described by Hosoi et al. [24], B16F10 melanoma cells, incubated overnight with phenol red-free DMEM containing 10% FBS and seeded on 6-well plate (2 × 10^5^ cells/well), were further incubated overnight. The cells were exposed to CM (10 *μ*L) for 72 h in the presence or absence of 500 nM *α*-MSH. The cells were washed with PBS and lysed with 250 *μ*L of 1 N NaOH containing 10% DMSO for 1 h at 70°C. The absorbance of the NaOH solution aliquot (200 *μ*L) at 490 nm was monitored using a microplate reader.

### 2.12. Cornified Envelope Formation Assay in Keratinocytes

The cornified envelope (CE) content, an index of corneocyte production, was determined as previously described [25]. Postconfluent HaCaT keratinocytes on 6-well plate were continually subjected to CM (10 *μ*L) for 5 days with medium changes every second day in FBS-free DMEM, harvested with a cell scraper, and homogenized in 2% SDS. After centrifuging at 5,000 g for 20 min, the precipitates were boiled in 2% SDS and 20 mM DTT for 1 h. The amounts of soluble crosslinked envelopes were determined by the absorbance at 310 nm using a microplate reader.

### 2.13. Antihyaluronidase Activity Assay

The antihyaluronidase activity of CMs was assessed by measuring a diminishment in hyaluronidase activity under its presence. The hyaluronidase activity was determined as previously described [26]. The mixture containing CM (10 *μ*L) and 20 *μ*L hyaluronidase solution (585 U/mL) was kept for 10 min at 37°C and added to the equal volume of HA solution (0.2 mg/mL). After the 45 min incubation, the 240 *μ*L of acidic albumin solution (79 mM acetic acid, 24 mM sodium acetate, and 0.1% BSA, pH 3.8 at 25°C) was added to the reaction mixture and was kept for 10 min at 25°C. The absorbance at 600 nm was measured at a microplate reader.

### 2.14. Antielastase Activity Assay

The antielastase activity of CMs was examined by measuring a diminishment in elastase activity under its presence. Elastase activity was assayed based upon the release of *p*-nitroaniline from STANA used as a synthetic substrate [27]. The reaction mixture containing 100 *μ*L of 0.2 M Tris buffer (pH 8.0) and CM (50 *μ*L) was preincubated with 100 *μ*L of 0.8 mM STANA for 20 min at 37°C, and the enzymatic reaction was begun with the addition of 50 *μ*L of 0.1 U/mL elastase. The absorbance at 410 nm was monitored using a microplate reader.

### 2.15. Procollagen Synthesis Assay

After the cultured NHDF cells on 6-well plate (5 × 10^5^ cells/well) were exposed to the CMs (10 *μ*L) for 48 h, the culture supernatants were prepared by centrifugation at 5,000 g for 10 min. The degree of collagen synthesis in the supernatants determined by measuring procollagen type-I C-peptide with PIP ELISA assay kit (Takara Bio Inc., Tokyo, Japan) following the manufacturer's protocol. The absorbance at 450 nm was monitored using a microplate reader.

### 2.16. Statistical Analyses

The results were shown as mean ± SD. The differences between experimental groups were analyzed utilizing one-way ANOVA subsequently with post hoc Tukey HSD test for multiple comparisons. In case of a *p* value less than 0.05, the difference was thought to be statistically significant.

## 3. Results

### 3.1. In Vitro Free Radical Scavenging Activities

Superoxide anion radical, which is one of the most frequently generated ROS in cells, is converted to other types of ROS, such as hydrogen peroxide and hydroxyl radical. Excessive superoxide radical anion, generated beyond the balancing capacities, is involved in several harmful biological processes, including protein denaturation and lipid peroxidation [28]. As shown in Figure 1(a), LP202, LF101, and LPP401 exhibited in vitro scavenging activities of 63.9 ± 4.4%, 86.7 ± 5.8%, and 92.7 ± 10.4%, respectively, against superoxide radical ion. Their scavenging activities were in the order of LPP401 ≥ LF101 > LP202, and MRS medium itself, used as a reference, was found to reveal a significantly lower scavenging activity against superoxide radical ion than the CMs (Figure 1(a)).

Nitric oxide (NO) is involved in various disease states, including inflammatory diseases, through the production of several reactive nitrogen species interacting with ROS. NO, acting as a major proinflammatory mediator, reacts with oxygen to form nitrite ions, and accordingly, extracellular nitrite ion level is regarded as an index of intracellular NO level. In the in vitro scavenging assays, LP202, LF101, and LPP401 scavenged the nitrite molecules at the percentages of 35.5 ± 1.0%, 35.8 ± 2.0%, and 56.8 ± 2.6%, respectively (Figure 1(b)). Their nitrite scavenging activities of the CMs were in the order of LPP401 > LF101≒LPP202. Likewise in the case of superoxide radical ion, MRS medium itself exerted a significantly lower scavenging activity against nitrite ions than the CMs (Figure 1(b)).

Collectively, the CMs have scavenging activities against superoxide radical and nitrite ions which might trigger oxidative/nitrosative stress inside cells.

### 3.2. Anti-Inflammatory Activities in LPS-Stimulated RAW264.7 Macrophages

When the cultured RAW264.7 macrophages were stimulated with LPS, the intracellular ROS and exogenous nitrite levels were elevated to 2.1- and 2.8-fold than those of the nonstimulated controls, respectively (Figures 2(a) and 2(b). As shown in Figure 2(a), LP202, LF101, and LPP401 attenuated the LPS-induced ROS levels to 81.5 ± 4.4%, 63.3 ± 0.8%, and 55.6 ± 2.1%, respectively, which gave rise to the order of LPP401 ≥ LF101 > LP202. As shown in Figure 2(b), LP202, LF101, and LPP401 attenuated the LPS-induced nitrite levels to 50.9 ± 11.4%, 35.8 ± 3.6%, and 30.6 ± 2.2%, respectively, in the order similar with the ROS measurement. AA, used as a positive control, gave rise to relatively high diminishments in both LPS-induced ROS and nitrite levels. As in Figure 2(c), it was confirmed that LPS treatment only and the CMs in the presence of LPS could not have any damaging influences on the viabilities of RAW264.7 macrophages. Taken together, these findings suggest that the CMs contain anti-inflammatory activities but in the order of LPP401 ≥ LF101 > LP202.

### 3.3. Skin Whitening Activities

Since tyrosinase is a key enzyme catalyzing a rate-limiting step of the melanin synthesis, it has been used as a well-known target for the development of skin whitening agents. Tyrosinase catalyzes the first two steps of melanin synthesis, the hydroxylation of L-tyrosine to L-DOPA and subsequently the oxidation of L-dopaquinone. The tyrosinase inhibitory activities of the CMs were measured and compared using L-DOPA as a substrate. As shown in Figure 3(a), LP202, LF101, and LPP401 exerted in vitro inhibitory effects against tyrosinase activity in the percentages of 79.1 ± 1.1%, 87.4 ± 1.4%, and 100 ± 0.6%, respectively. Their inhibitory activities were found to be in the order of LPP401 > LF101 ≥ LP202. MRS medium itself displayed a significantly low inhibitory activity against tyrosinase.

Effects of the CMs were measured and compared on melanin production in cultured B16F10 melanoma cells. *α*-MSH was identified to increase the melanin content to 1.7-fold (Figure 3(b)). As shown in Figure 3(b), LP202, LF101, and LPP401 attenuated the *α*-MSH-induced melanin levels to 71.9 ± 2.3%, 42.5 ± 4.1%, and 39.5 ± 3.4%, respectively, which were in the order of LPP401≒LF101 > LP202. Arbutin (AR), a positive control, and MRS medium itself could diminish the *α*-MSH-induced melanin levels to 76.7 ± 2.7% and 89.2 ± 3.7%, respectively.  Figure 3(c) confirms that *α*-MSH only and the CMs in the presence of *α*-MSH had no cytotoxic effects on the viabilities of cultured B16F10 melanoma cells.

Collectively, these findings suggest that the CMs possess skin whitening activities, but in the overall order of LPP401 > LF101 ≥ LP202, plausibly through the suppression of melanin synthesis via the inhibition of tyrosinase activity.

### 3.4. Skin Barrier Function-Improving Activities

The skin barrier function, located in the stratum corneum, is to protect the body from excessive transepidermal water loss and to prevent the penetration of compounds, such as chemicals, infectious agents, systemic toxicity, and allergens, into the body via the epidermis. If the terminally differentiated keratinocytes in the cornified layer of the stratum corneum, so called corneocytes, responsible for skin barrier function, are not sufficiently and suitably formed, undesirable substances are more easily rendered to the skin. Effects of LP202, LF101, and LPP401 were evaluated on the formation of corneocytes in HaCaT keratinocytes based on the quantitation of cornified envelopes. In Figure 4(a), LP202, LF101, and LPP401 were able to augment the cornified envelope contents to 1.2-, 1.6-, and 2.1-fold, respectively. However, MRS medium itself showed no enhancing effect in the levels of cornified envelopes. As shown in Figure 4(b), it was convinced that the CMs did not exert toxic effects on the viabilities of HaCaT keratinocytes used. In brief, LP202, LF101, and LPP401 have skin barrier function-improving properties, but in the order of LPP401 > LF101 > LP202.

### 3.5. Antihyaluronidase and Antielastase Activities

The age-dependent loss of hyaluronan and elastin, due to their insufficient production and increased degradation, leads to alterations in the skin homeostasis, which results in the various kinds of skin problems and disorders. The inhibition of hyaluronidase and elastase activities, responsible for the degradations of hyaluronan and elastin, respectively, may be useful for restoring and maintaining the homeostasis of the skin, subsequently improving dysfunction and reducing various age-related disorders. As shown in Figure 5(a), LP202, LF101, and LPP401 showed inhibitory activities against hyaluronidase at the percentages of 10.8 ± 1.4%, 9.1 ± 1.8%, and 21.8 ± 5.8%, respectively, which were in the order of LPP401 > LP202 ≥ LF101. As shown in Figure 5(b), LP202, LF101, and LPP401 showed inhibitory activities against elastase at the percentages of 17.2 ± 1.6%, 15.1 ± 2.0%, and 19.0 ± 1.6%, respectively, which were in the order of LPP401 ≥ LP202 > LF101. Taken together, LP202, LF101, and LPP401 contain both antihyaluronidase and antielastase activities. However, LP401 displays higher inhibitory activities against both the enzyme activities than LP202 and LF101.

### 3.6. Collagen Production-Promoting Activities

Collagen is a main structural protein in the extracellular matrix, which is responsible for structure, strength, texture, elasticity, and resilience in skins. Collagen production declines with age and exposure to UV radiation and environmental stressors including pollution and smoking, which contributes to sagging and wrinkles as the visible signs of skin aging. In cultured NHDF cells, the effects of CMs were evaluated and compared on the production of procollagen type 1, the precursor of collagen type 1 as the major collagen in skins, through the quantitation of C-peptide using PIP EIA kit. As shown in Figure 6(a), LP202, LF101, and LPP401 augmented the C-peptide levels to 1.06-, 1.45-, and 1.43-fold, compared with the control level. MRS medium itself was measured to have no modulating effect on the C-peptide levels (Figure 6(a)). The CMs, at the used concentration, were observed to be nontoxic on the viabilities of the NHDF cells (Figure 6(b)). Collectively, LF101 and LPP401, but not LP202, are capable of enhancing the collagen production with similar degrees in fibroblasts, further supporting their skin antiaging abilities.

## 4. Discussion

It is generally accepted that the diverse members of the genus *Lactobacillus* and even the different subspecies strains within the same *Lactobacillus* species can possess dissimilar physiological functions in humans. To date, it has been ascertained that *L. plantarum*, *L. fermentum*, and *L. paraplantarum* possess a broad variety of health beneficial properties, including skin beneficial properties relating to this work. *L. plantarum* HY7714 rescues UV-B-reduced procollagen expression through the inhibition of UV-B-induced matrix metalloproteinase-1 expression in human dermal fibroblasts, and its oral administration inhibits the number, depth, and area of wrinkles in the hairless mouse skin, implying that it is a skin antiphotoaging agent [7]. *L. plantarum* HY7714 enhances skin hydration, reduces wrinkles, and improves skin elasticity, hinting its skin antiaging benefit [8]. Oral administration of heat-killed *L. plantarum* L-137 suppresses the loss of water content in the stratum corneum in hairless mice [9]. The treatment of primary epidermal cells with heat-killed *L. plantarum* L-137 augments the production of hyaluronan, which suggests its usefulness for the improvement of skin functions, such as moisture retention, by enhancing hyaluronan production [9]. The cell-free supernatant and the protein-rich fraction from *L. plantarum* USM8613 inhibit staphyloxanthin biosynthesis, reduce the cell number of *S. aureus*, and reduce biofilm thickness in *S. aureus*-infected porcine skins [10]. It also exerts wound healing properties via the direct inhibition of *S. aureus* and promotes innate immunity in rats, in which the expression of *β*-defensin is upregulated through the production of cytokines and chemokines during wound recovery [10]. Lipoteichoic acid isolated from *L. plantarum* was shown to be used as a cosmetic whitening agent through the inhibition of melanogenesis via its suppressive effect on the cellular activity of tyrosinase and the expression of tyrosinase family members [11]. An *L. plantarum*-GMNL6 extract enhances the collagen synthesis and reduces the melanin synthesis, the biofilm of *S. aureus*, and the proliferation of *Cutibacterium acnes* via improving the human skin microbiota, which proposes its regulatory effects on human skin health [29].

A variety of strains belonging to the species *L. fermentum* have gained a particular attention due to their novel health beneficial efficacies assessed in recent years. *L. fermentum* JX306 attenuates D-galactose-induced oxidative stress of mice by decreasing malondialdehyde levels, enhancing glutathione peroxidase activity and total antioxygenic capacity in the serum, kidney, and liver, and upregulating the transcriptional levels of antioxidant enzyme genes in the liver [12]. *L. fermentum* PC1 has a treatment potential against rheumatoid arthritis in the murine model of collagen-induced arthritis through the attenuation of proinflammatory cytokine IL-12 and the augmentation of anti-inflammatory cytokines IL-4 and IL-10 [30]. Dietary *L. fermentum* V3 was identified to ameliorate colon cancer progression by modulating the gut microbiota community [31]. *L. fermentum* TKSN, in combination with nicotinamide mononucleotide, improves skin damages caused by UV-B radiation in mice through the activation of AMP-activated protein kinase signaling pathway, which implies the preventing and treating skin photoaging [14].

Although *L. paraplanatrum*, as a relatively recent member of the genus *Lactobacillus*, has been less studied, it is known to have some peculiar efficacies, including women-specific benefits. *L. paraplantarum* L-ZS9, isolated from fermented sausage, and produces class II bacteriocins to suppress the growth of pathogenic bacteria [32]. *L. paraplantarum*, isolated from fermented dates in Saudi Arabia, was verified to possess the antifungal, probiotic, and antioxidant properties [16]. *L. paraplantarum* SC61, isolated from a Korean fermented food, displays antioxidant activity, including DPPH radical scavenging, *β*-carotene bleaching inhibition, reducing power, superoxide anion scavenging, ABTS^+^ scavenging activity, and immunostimulatory activity [17]. A high molecular weight exopolysaccharide from *L. paraplantarum* BGCG11 (EPS CG11) was identified to possess antihyperalgesic and antiedematous effects, related to the suppression of inflammatory response, in the rat model of inflammation induced by carrageenan in hind paw [18]. It also exhibits immunosuppressive properties in the peritonitis model induced by carrageenan related to the suppression of inflammatory response [18].

This work has been performed to evaluate and compare the cosmetic potentials of the three *Lactobacillus* strains, *L. plantarum* SB202, *L. fermentum* SB101, and *L. paraplantarum* SB401, which are indigenous to the skins of Korean people, in the search for more favorable probiotic resource(s) to be utilized for the manufacture of novel functional cosmetics. Based on the 16S rDNA nucleotide sequences, *L. plantarum* SB202 and *L. paraplantarum* SB401 were identified to share the nucleotide sequence homology of 99%, and each of them shares the reduced nucleotide sequence homology of 91% with *L. fermentum* SB101 (data not shown). Among the three *Lactobacillus* strains, these homologies reveal highly similarity between *L. plantarum* SB202 and *L. paraplantarum* SB401 on the genetic and evolutionary basis. The cosmetic potentials of the *Lactobacillus* strains, comparatively assessed in this work, are summarized in Table 1. The CMs, individually prepared from the cultures of the three *Lactobacillus* cells, were convinced to have the tested cosmetic potentials, such as in vitro free radical scavenging, anti-inflammatory, skin whitening, barrier function-improving, and anti-aging properties, though there were more or less differences between them. In the in vitro scavenging against superoxide radical ion, LF101 and LP401 exerted higher activities than LP202, and in the in vitro scavenging against nitrite ion, LPP401 gave rise to much higher scavenging activity than LP202 and LF101. In the LPS-stimulated RAW264.7 inflammatory model, both LF101 and LPP401 displayed higher attenuating activities on the LPS-induced ROS and nitrite levels than LP202, which were in the similar patterns with their superoxide radical ion scavenging activities. In the skin whitening activity assay, all of the three CMs displayed significantly high inhibitory activities against tyrosinase, and LF101 and LPP401 showed markedly higher suppressive activities on the *α*-MSH-induced melanin contents than LP202 in B16F10 melanoma cells. In the assays of cornified envelope formation to estimate skin barrier function in HaCaT keratinocytes, LP202 displayed no modulating activity on the cornfield envelope formation, but LP401 exerted higher enhancing activity than LF101. The antihyaluronidase activity of LPP401 was higher than those of LP202 and LF101, but the three CMs exerted the similar antielastase activities. LF101 and LPP401, but not LP202, appeared to upregulate the production procollagen type 1. These findings indicate that LPP401 is supposed to possess more favorable skin antiaging property among the three CMs.

Until recently, probiotic bacteria, including the genera *Lactobacillus* and *Bifidobacterium*, have verified to produce diverse therapeutic compounds such as amino acid metabolites, vitamins (folate, vitamins B1, B2, B6, B9, and B12), bacteriocins, diacetyl, hyaluronic acid, exopolysaccharides, fructooligosaccharides (inulin, levan), enzymes (amylase, superoxide dismutase, catalase, sphingomyelinase), immunomodulatory compounds, short-chain fatty acids (lactic acid, butyric acid, propionic acid, acetic acid), lipoteichoic acid, and peptidoglycan [33, 34]. However, the possible action mechanisms by which the known compounds exhibit skin beneficial properties as cell-free CM ingredients are largely unknown. In this work, comparatively evaluating the skin beneficial properties of the three *Lactobacillus* strains newly isolated from the healthy skins of Koreans, the responsible components of the cell-free CMs have not been analyzed yet. Studies on the differences in therapeutic components and accompanying action mechanisms between the three *Lactobacillus* strains would be possibly done in the continuing works. In this work, the cell-free CMs of the three *Lactobacillus* strains of human skin origin, isolated and partly characterized through this work, appeared to be nontoxic to RAW264.7 murine macrophages, B16F10 murine melanoma cells, HaCaT keratinocytes, and normal human dermal fibroblast (NHDF) cells, which in part supports their safe topical application.

Based on the overall cosmetic potentials of the CMs from the three skin *Lactobacillus* isolates, *L. paraplantarum* SB401 has been thought to be more desirable probiotic resource, then followed by *L. fermentum* SB101, which can be applied in the manufacture of novel functional cosmetics. However, further mechanistic approaches will be needed for better application performance.

## 5. Conclusion

In conclusion, the conditioned mediums, prepared from the cultures of three *Lactobacillus* strains indigenous to Korean skins, *L. plantarum* SB202, *L. fermentum* SB101, and *L. paraplantarum* SB401, have been assessed to have skin beneficial properties such as in vitro free radical scavenging, anti-inflammatory, whitening, barrier function-improving, and antiaging activities. Although there were more or less variable among the conditioned mediums of the three *Lactobacillus* strains, which were dependent on the individual skin beneficial characteristics, the conditioned medium of *L. paraplantarum* SB401, followed by that of *L. fermentum* SB101, appeared to be more appropriate as a probiotic candidate applicable to cosmetic industry, based upon the overall skin beneficial characteristics evaluated in this work.

## Figures and Tables

**Figure 1:** The in vitro scavenging activities of the three conditioned media (LP202, LF101, LPP401) on superoxide radical (a) and nitrite (b) ions. MRS broth (MRS) is the liquid medium used for the *Lactobacillus* growth. The data represent the percentage of the anion scavenging. ^∗∗∗^*p* < 0.001 vs. MRS.

**Figure 2:** The effects of LP202, LF101, and LPP401 on the LPS-induced levels of ROS (a) and nitrite ions (b) and the cell viability (c) in LPS-stimulated RAW264.7 murine macrophages. Ascorbic acid (AA) was used as a positive control. ^###^*p* < 0.001 versus non-LPS control. ^∗∗^*p* < 0.01; ^∗∗∗^*p* < 0.001 versus the nontreated control (LPS treatment alone).

**Figure 3:** The effects of LP202, LF101, and LPP401 on in vitro tyrosinase activity (a) and the *α*-MSH-induced melanin contents (b) and the cell viability (c) in *α*-MSH-stimulated B16F10 murine melanoma cells. In (a), purified mushroom tyrosinase and L-DOPA were used as an enzymes source and a substrate, respectively. Arbutin (AR) was used as a positive control. ^###^*p* < 0.001 versus non-LPS control. ^∗∗∗^*p* < 0.001 vs. MRS (in (a)) or the nontreated control (LPS treatment alone) (in (b)).

**Figure 4:** The effects of LP202, LF101, and LPP401 on the cornified envelope formation (a) and the cell viability (b) in HaCaT keratinocytes. In (a), the relative percentage of cornified envelope formation was calculated by considering the control value as 100. ^∗∗∗^*p* < 0.001 vs. the nontreated control.

**Figure 5:** The inhibitory effects of LP202, LF101, and LPP401 on hyaluronidase (a) and elastase (b) activities. In (a), hyaluronan was used as a substrate of purified hyaluronidase. In (b), *N*-succinyl-Ala-Ala-Ala-*p*-nitroanilide was used as a chromogenic substrate of elastase. The data represent the percentage of enzyme activity inhibition. ^∗^*p* < 0.05; ^∗∗^*p* < 0.01; ^∗∗∗^*p* < 0.001 vs. MRS.

**Figure 6:** The effects of LP202, LF101, and LPP401 on the level of procollagen type I C-peptide (a) and the cell viability (b) in normal human dermal fibroblast (NHDF) cells. Ascorbic acid (AA) was used as a positive control. ^∗∗^*p* < 0.01 versus the nontreated control.

**Table 1:** Summary on the skin beneficial properties of the three conditioned mediums.

Skin beneficial activities	Relative activities^∗^		
	LP202	LF101	LPP401
In vitro free radical scavenging activities			
Superoxide radical ion scavenging	++	+++	+++
Nitrite ion scavenging	++	++	+++
Anti-inflammatory activities in macrophages			
Attenuation of LPS-induced ROS	+	+++	+++
Attenuation of LPS-induced NO	++	+++	+++
Skin whitening activities			
Antityrosinase activity	++	++	+++
Attenuation of melanin in melanoma cells	+	+++	+++
Skin barrier function-enhancing activity			
Enhancement of cornified envelope formation in keratinocytes	+	++	+++
Antiaging enzyme activities			
Antihyaluronidase activity	+	+	+++
Antielastase activity	+++	+++	+++
Collagen production-promoting activity			
Enhancement of collagen synthesis in fibroblasts	—	++	++

^∗^+: weak; ++: moderate; +++: strong; –: no activity.

## Data Availability

The data used to support the findings of this work are available to other researchers from the corresponding author upon request.
